# Inhibition of *Staphylococcus aureus* Efflux Pump by O-Eugenol and Its Toxicity in *Drosophila melanogaster* Animal Model

**DOI:** 10.1155/2022/1440996

**Published:** 2022-07-19

**Authors:** Nair Silva Macêdo, Zildene de Sousa Silveira, Paula Patrícia Marques Cordeiro, Henrique Douglas Melo Coutinho, José Pinto Siqueira Júnior, Lucindo José Quintans Júnior, Abolghasem Siyadatpanah, Bonglee Kim, Francisco Assis Bezerra da Cunha, Márcia Vanusa da Silva

**Affiliations:** ^1^Graduate Program in Biological Sciences-PPGCB, Federal University of Pernambuco-UFPE, Recife, PE, Brazil; ^2^Laboratory of Semi-Arid Bioprospecting (LABSEMA), Regional University of Cariri-URCA, Crato, CE, Brazil; ^3^Laboratory of Microbiology and Molecular Biology (LMBM), Regional University of Cariri-URCA, Crato, CE, Brazil; ^4^Laboratory of Microorganism Genetics (LGM), Department of Molecular Biology, Federal University of Paraiba-UFPB, Brazil; ^5^Laboratory of Neuroscience and Pharmacological Tests-LANEF, Federal University of Sergipe, Aracaju, SE, Brazil; ^6^Ferdows Paramedical School, Birjand University of Medical Sciences, Birjand, Iran; ^7^Department of Pathology, College of Korean Medicine, Kyung Hee University, Seoul 02447, Republic of Korea

## Abstract

**Background:**

Efflux pumps are transmembrane proteins that expel drugs out of a bacterial cell contributing to microorganism drug resistance. Several studies addressing the use of natural products with medicinal properties have intensified given the above. Thus, the aim of the present study was to investigate the antibacterial activity and the O-eugenol potential in *Staphylococcus aureus* resistance reversal by efflux pump inhibition, as well as to evaluate its toxicity in the *Drosophila melanogaster* arthropod model. The broth microdilution method was used to determine the minimum inhibitory concentration (MIC) and the O-eugenol efflux pump inhibition. For the *D. melanogaster* toxicity assays, mortality and locomotor system damage were performed using the fumigation method.

**Results:**

O-eugenol presented a MIC of 1024 *μ*g/mL against *S. aureus*. The association of this compound with the antibiotic tetracycline demonstrated a synergistic effect (*p* < 0.0001), this also being observed when the antibiotic was associated with ethidium bromide (*p* < 0.0001); thus, these results may be attributable to an efflux pump inhibition. The *D. melanogaster* mortality and geotaxis assays revealed the compound is toxic, with an EC_50_ of 18 *μ*g/mL within 48 hours of exposure.

**Conclusions:**

While we can conclude that the tested product has an efflux pump inhibitory effect, further studies are needed to elucidate its mechanisms of action, in addition to assays using other strains to verify whether the substance has the same inhibitory effect.

## 1. Introduction

Efflux pumps are one of the resistance mechanisms used by pathogenic microorganisms, this being characterized by actively expelling drugs from the bacterial cell, thus collaborating with the appearance of multidrug-resistant (MDR) phenotypes in strains with clinical interest [1, 2], where the genes that code for efflux pumps can be located on the chromosomes or plasmids of these microorganisms [3].

*Staphylococcus aureus* is among these infectious pathogens, being easily contracted by humans due to its ample capacity to synthesize extracellular toxins, as well as for presenting known virulence factors such as staphylococcal enterotoxins [4]. Moreover, *S. aureus* is able to acquire resistance to a variety of antimicrobial agents [5]. The IS-58 strain, which carries the TetK efflux pump, is among the strains of clinical interest [6]. This pump has the efflux protein that confers resistance to tetracyclines and is part of the major facilitator superfamily (MFS) family that uses energy from a proton gradient to extrude the antibiotic [7].

Therefore, the search for new natural bacterial resistance modifiers has been intensified, aiming at the reintroduction of ineffective therapeutic antibiotics in clinical practice [8]. Thus, some phytochemicals can act as adjuvants, inhibiting target-modifying and drug-degrading enzymes, or as inhibitors of efflux pumps [9]. Phenolic compounds stand out among these phytochemicals given their several bioactivities, such as antioxidant, anti-inflammatory, antiallergic, antithrombotic, antimicrobial, and antineoplastic activity [10, 11]. O-eugenol (2-allyl-6-methoxyphenol) is defined as a phenolic derivative and has a hydroxyl group moved to the carbon that is situated between the methoxy and allyl groups [12, 13].

While many of these phenolic compounds can present antimicrobial activities, these can have a high toxicity and be harmful to eukaryotic cells [14]. *Drosophila melanogaster*, an organism that has a low maintenance cost in the laboratory and a short reproductive cycle, in addition to being highly sensitive to the presence of toxic substances at minimal concentrations, is one of the models used to assess the toxicity of these compounds [15, 16].

With this in mind, the objective of the present study was to investigate the antibacterial activity of the isolated O-eugenol compound and its potential for reversing *Staphylococcus aureus* resistance by efflux pump inhibition, as well as to evaluate its toxicity in the *D. melanogaster* arthropod model.

## 2. Materials and Methods

### 2.1. Culture Media and Microbial Strains

The IS-58 *Staphylococcus aureus* strain, endowed with the PT181 plasmid carrying the TetK, tetracycline efflux protein, gene was used. The strain was provided by Prof. S. Gibbons (University of London). The bacteria were kept in blood agar base supplements with the antibiotic tetracycline to maintain the plasmid (Laboratórios Difco Ltda., Brazil) and then transferred and kept in glycerol -80°C. Heart Infusion Agar (HIA, Difco laboratorises Ltda.), prepared according to the manufacturer, and 10% Brain Heart Infusion (BHI Acumedia Manufacturers Inc.) were used as the culture media in the assays.

### 2.2. Substances

Tetracycline was the antibiotic used, this being specific to the strain carrying the TetK pump. The antibiotic and O-eugenol were diluted in dimethyl sulfoxide (DMSO), then in sterile water. Chlorpromazine and ethidium bromide (EtBr) were dissolved in distilled sterile water; carbonyl cyanide m-chlorophenylhydrazone (CCCP) was dissolved in methanol/water (1 : 1, *v*/*v*). All substances were diluted to a concentration of 1024 *μ*g/mL, stored at 20°C, and protected from light. All substances were purchased from Sigma-Aldrich Brazil, except chlorpromazine, which was purchased from a commercial pharmacy.

### 2.3. Determination of the Minimum Inhibitory Concentration (MIC)

MIC is defined as the lowest concentration that inhibits the visible growth of a microorganism [17]. The MIC was determined for O-eugenol and tetracycline using the broth microdilution method [18]. The stock strains were sprayed in HIA medium and incubated at 37°C for a period of 24 hours. The inoculants were prepared in test tubes containing 3 mL of sterile saline solution, these being compared to the 0.5 McFarland scale which corresponds to 10^6^ CFU (colony forming units). Then, Eppendorfs® containing 1.440 *μ*L of the BHI liquid culture medium and 160 *μ*L of the bacterial inoculum were prepared, forming a final volume of 1.6 mL. After mixing 1,140 *μ*L of BHI plus 160 *μ*L of the inoculum (~10^5^ CFU/mL), the inoculum was diluted 10 times. Subsequently, microdilution plates were filled, with rows 7 and 8 being growth controls and rows 9 and 10 sterility controls. Microdilution was performed with O-eugenol (100 *μ*L) in the first 6 rows, where concentrations ranged from 512 *μ*g/mL to 4 *μ*g/mL. The plates were incubated in a bacteriological incubator at 37°C for 24 hours. The assay was finished by adding 20 *μ*L of resazurin [19], a redox dye to evaluate the presence of cell metabolism, with the color change of the medium from blue to red being an indicative of the bacterial growth [20].

### 2.4. Antibiotic Modulatory Effect and Efflux Pump Inhibition Evaluation by an Ethidium Bromide (EtBr) Modulatory Effect

For this, Eppendorfs® were filled with 160 *μ*L of the inoculum, O-eugenol at a subinhibitory concentration (MIC/8), and completed with BHI until reaching a volume of 1.6 mL. A modulation control was prepared with 160 *μ*L of the inoculum and 1.440 *μ*L of BHI without the O-eugenol, and 100 *μ*L of the antibiotic was sequentially diluted. Microdilution plates were then filled, where rows G and H were reserved for bacterial growth controls. Sterility controls were performed on separate plates. Subsequently, a microdilution was performed with the antibiotic (100 *μ*L) to assess the modulatory effect of the antibiotic, with concentrations ranging between 0.25 and 512 *μ*g/mL.

The efflux pump inhibition assays were performed by evaluating the decrease in the MIC of ethidium bromide, since the efflux pumps are the only mechanism responsible for the extrusion of EtBr. Microdilution was performed with 100 *μ*L of EtBr for the inhibitory evaluation of the efflux pump. A modulation control was prepared with 160 *μ*L of the inoculum and 1.440 *μ*L of BHI without the O-eugenol, and 100 *μ*L of the EtBr was sequentially diluted. Concentrations ranged from 512 *μ*g/mL to 0.25 *μ*g/mL [21]. After 24 h, readings were performed by adding 20 *μ*L of resazurin [19].

### 2.5. *Drosophila melanogaster* Stock

*D. melanogaster* (Harwich strain) was obtained from the National Species Stock Center, Bowling Green, OH. The flies were cultivated in 340 mL glass bottles grown with the medium containing: 83% corn mass, 4% sugar, 4% lyophilized milk, 4% soy bran, 4% wheat bran or oats, and 1% salt. 1 g of Nipagin (Methylparaben) was added when cooking the mixture. Following a cooling period in the growth flasks, 1 mL of a solution containing *Saccharomyces cerevisiae* was added to the flask. The flies were grown in photoperiod BOD greenhouses at a temperature of 25°C ± 1°C and 60% relative humidity.

### 2.6. Mortality Assays

*Drosophila melanogaster* is widely used to assay in vivo toxicity, because through its sensitivity to harmful substances in minimal concentrations, it is an important model to assess the toxic activity of these substances [22]. The fumigation bioassay methodology was used to evaluate the O-eugenol toxicity, where adult flies (males and females aged approximately 3 to 5 days) were placed in 130 mL flasks in multiples of 20, previously prepared with 1 mL of a sucrose solution in distilled water, at a concentration of 20%, allowing the flies to feed *ad libitum*. This solution was soaked in a paper and placed on the bottom of the glass, while the glass cover had a filter paper. The control was prepared with 20 *μ*L of acetone. The compound O-eugenol was diluted in acetone according to its molecular weight obtaining a stock solution of 213.6 *μ*g/mL. After that, volumes of 20, 10, and 5 *μ*L of this stock solution were withdrawn, resulting in final concentrations of 33, 16, and 8 *μ*g/mL air using 130 mL air bottles, respectively. All bioassays were conducted in a BOD-type greenhouse with a 12-hour light and dark cycle, with the temperature controlled at 25°C ± 1°C and 60% relative humidity. The tests were performed in triplicates, and mortality rate readings were made at 3, 6, 12, 24, 36, and 48 hours [15].

### 2.7. Negative Geotaxis Assay

Damage to the locomotor system was determined by a negative geotaxis test, which consists of counting the number of flies that rise above 3 cm in the glass column of the experiment itself in a 5-second time interval, this being repeated 2 times at 1-minute intervals [23]. This test was performed every 3, 6, 12, 24, 36, and 48 hours. The results were presented as the mean time (s) ± SE obtained from two independent experiments.

### 2.8. Statistical Analysis

Statistical analysis for the microbiological tests was performed using a two-way ANOVA followed by Bonferroni's *post hoc* test, using the GraphPad Prism 7.0 software. For the toxicity data analysis, a two-way ANOVA followed by Tukey's multiple comparisons test was performed. No statistical differences were observed with the same concentration as a function of time.

## 3. Results

### 3.1. Efflux Pump Inhibition by Antibiotic and Ethidium Bromide MIC Reductions

O-eugenol demonstrated a MIC of 1024 *μ*g/mL against the IS-58 *S. aureus* strain. The association between O-eugenol and the antibiotic tetracycline revealed a reduction in the antibiotic's MIC, indicating a potentiation of antibiotic activity, as observed in Figure 1. When the antibiotic was tested in association with standard inhibitors at subinhibitory concentrations, the MIC values for chlorpromazine did not differ from the antibiotic control, whereas the MIC for CCCP presented a marked synergism. CCCP and chlorpromazine are standard efflux pump inhibitors, but have no direct effect on the efflux pump. They act inhibiting by modifying the transmembrane electrochemical potential of the bacteria [24].

Table 1 represents the association values of the specific antibiotic tetracycline and EtBr with standard inhibitors (CCCP and chlorpromazine). In terms of efflux pump inhibitory assays based on the reduction of the ethidium bromide MIC, its association with O-eugenol (MIC/8) presented a decrease in the MIC of EtBr from 32 to 16 *μ*g/mL, as seen in Table 1, this being characterized as a synergistic action.  Figure 2 shows that similar results were observed for the standard inhibitors.

### 3.2. *Drosophila melanogaster* Toxicity

O-eugenol obtained an EC_50_ of 18 *μ*g/mL within 48 hours of exposure. The results obtained with the *Drosophila melanogaster* toxicity test showed that O-eugenol presented moderate toxicity at the 33 *μ*g/mL concentration after 3 hours of exposure, with the mortality rate increasing following the hours of exposure (Figure 3). Significant mortality was observed after 36 hours of exposure to the compound for the 16 *μ*g/mL concentration (Figure 3).

In the negative geotaxis assays where possible damage to the locomotor apparatus is verified, a significant locomotor deficit was observed in the flies (*p* < 0.0001) at the 33 *μ*g/mL air concentration at a 3-hour exposure period when compared to the control (Figure 4). This effect was intensified over the following hours of exposure, and a marked damage to the locomotor apparatus was observed at the 24-hour reading, as the alive flies showed difficulty in locomotion (Figure 4).

## 4. Discussion

The MIC is defined as the lowest concentration capable of completely inhibiting microbial growth [25] and thus is considered clinically irrelevant when it is insufficient to inhibit bacterial growth. There are no studies evaluating the antimicrobial activity of O-eugenol on bacterial strains in the literature. Furthermore, in the present study, the antibacterial activity of O-eugenol on the IS-58 strain of *S. aureus* was not verified. The phenolic compounds caffeic acid and gallic acid demonstrated a MIC of 1024 *μ*g/mL for the IS-58 *S. aureus* strain [26].

However, other phenolic compounds have already shown antibacterial activity, as the results observed in experiments with quercetin, which showed antimicrobial activity on *S. aureus*, obtaining a MIC value of 6.25 *μ*g/mL [27]. A MIC value considered to be relevant was also found in assays with eugenol against the *S. aureus* ATCC 25923 strain, with this MIC value being 256 *μ*g/mL [28].

In addition to the antimicrobial action of isolated phenolic compounds, the action of plant extracts with high total phenolic and flavonoid contents has also been reported in the literature, for example, the *Corymbia ficifolia* (Eucalyptus) extract with the following compounds, gentisic acid, chlorogenic acids, p-coumaric, hyperoside, isoquercitrin, rutin, and quercitrin, presented an antibacterial activity against the *S. aureus* strain with a MIC value of 20 *μ*g/mL [29].

Although O-eugenol did not show direct antibacterial activity against the IS-58 strain of *S. aureus*, synergism was observed when associated with the antibiotic tetracycline, as shown in Figure 1. Assays using quercetin and its morin isomer showed potential to reduce 3 to 16 times the MIC of tetracycline on methicillin-resistant *S. aureus* strains (MSSA-MSRA) [30].

Efflux pumps are associated with pathogenic resistance phenotypes, thus representing an important threat to the effective treatment of diseases triggered by Gram-negative and Gram-positive bacteria [31]. In the IS-58 strain of *S. aureus*, the TetK efflux pump is responsible for the mechanism of bacterial resistance to tetracycline, which acts by extruding the antibiotic out of the bacterial cell [32]. By this fact, it is extremely important to identify and produce efflux pump inhibitors (EPIs) from natural sources, such as plants which have secondary bioactive metabolites [33]. These EPIs can act by triggering an energy depletion process, by preventing binding to ATP or altering the proton gradient [34].

Although our results show that there was no direct antibacterial activity on the IS-58 strain of *S. aureus*, synergism was observed when O-eugenol was associated with the antibiotic and EtBr, decreasing their MICs, indicating that the compound acts on the resistance mechanism characterized as active efflux, which is promoted by efflux pumps that actively expel EtBr to the outside of the cell, decreasing its toxicity on bacterial cells [35].

The use of ethidium bromide as a substrate for efflux pumps is well described in the literature, and as shown in Figure 2, O-eugenol presented a behavior similar to that of standard inhibitors, pointing to a similar pump inhibitory mechanism against the analyzed strain. The TetK efflux pump present in the IS-58 strain of *S. aureus* is responsible for therapeutic resistance to antibiotics of the tetracycline class. To combat bacterial resistance, a wide range of studies has been conducted to verify whether natural products act as adjuvants to antibiotics. In this perspective, products obtained from plant sources, rich in phytochemicals such as phenolic compounds, flavonoids, tannins, and phenolic acids, can act synergistically when associated with antibiotics against *S. aureus* strains that carry efflux pumps. It is important to note that there are no studies reporting the inhibitory effects of O-eugenol on the IS-58 (TetK) pump in *S. aureus*, with this study being the first to report this activity. However, there are other studies in the literature analyzing other phenolic compounds as possible efflux pump inhibitors, for example, assays performed with caffeic acid and gallic acid. Caffeic acid when combined with ethidium bromide reduced the MIC against strains carrying the TetK, MrsA, and NorA pumps; however, it only inhibited the action of the *S. aureus* MrsA and NorA efflux pumps. On the other hand, gallic acid reduced the MIC of ethidium bromide against *S. aureus* strains that had the TetK, MrsA, and NorA pumps; however, bacterial resistance reversal by efflux pump inhibition was only observed in the strain with the NorA pump [26].

Another study evaluates the antibacterial activity of natural products on *S. aureus* strains carrying the TetK efflux protein. Recent research has evaluated the potential of two natural compounds, *α*-bisabolol and *β*-cyclodextrin, and it was observed that these compounds when associated with the antibiotic tetracycline showed synergistic action, in other words, reduced the MIC of tetracycline [36].

Another study in the literature demonstrates the antibacterial effect of menadione (vitamin K) on this same strain (IS-58) of *S. aureus* with an MIC value of 64 *μ*g/mL. And when menadione was associated with ethidium bromide, there was a reduction in the MIC of BrEt, indicating inhibition of the efflux pump mechanism [34]. The essential oil from *Chenopodium ambrosioides* L. leaves also reduced the MIC of ethidium bromide, demonstrating inhibition on the TetK efflux pump [37].

Experiments using tannic acid showed its potential to decrease the MIC of antibiotics and ethidium bromide against *S. aureus* strains carrying MrsA and TetK efflux pumps, indicating this substance can inhibit the resistance mechanisms to these antibiotics [31]. The antimicrobial effects of phenolic acids are attributable to their chemical structure, especially to the length of the saturated chain, and position and number of substitutions in the benzene ring of the nucleus [38].

An analysis of twelve flavonoids showed that four of these (naringenin, phloretin, diosmetin, and myricitrin) decreased the MIC of the antibiotic norfloxacin from 128 *μ*g/mL to 32 *μ*g/mL, this equating to a fourfold reduction, while hesperetin resulted in a reduction from 128 *μ*g/mL to 8 *μ*g/mL, a sixteenfold decrease, against *S. aureus* SA-1199B. For association assays with ethidium bromide, naringenin stood out by decreasing the MIC of EtBr from 32 *μ*g/mL to 8 *μ*g/mL, a fourfold reduction [39].

The results obtained in this study suggest that O-eugenol may present antibacterial effect modifier activity; in other words, decreasing the antibiotic concentration required to suppress the growth of bacterial pathogens such as *S. aureus*, when used as adjuvants in antibiotic therapy against these pathogens. Recent reports have evidenced that the association of some terpenes with conventional antibiotics resulted in increased antibiotic activity, reversing the antibiotic resistance observed experimentally [40].

The bioactivities of a plant or an isolated compound are considered excellent when toxicity or adverse events considered lethal in experimental models are not observed. For this reason, toxicity evaluation studies are of paramount importance [14]. Invertebrate models, such as *D. melanogaster*, have been widely used in studies to assess the toxicity and genotoxicity of natural products since this model has many signaling pathways similar to those of humans, in addition to having drug target homology with vertebrate models, such as rodents and other small mammals [41]. There are no reports of studies in the literature evaluating the toxicity of the O-eugenol compound on the *D. melanogaster* arthropod model, this study being the first to report this effect.

*D. melanogaster* is characterized as an alternative eukaryotic model that has been widely used to verify the toxicity of substances due to aspects that favor its use, namely, its high sensitivity to low concentrations of substances, easy maintenance in the laboratory, short reproductive cycle, and high number of offspring [42]. In the literature, there are several studies that associate the antibacterial activity and toxicity of substances using *D. melanogaster* as a result of the factors mentioned above.

The fruit fly has been used to analyze the toxicity of several compounds, including eugenol and isoeugenol, which showed a high toxicity against *D. melanogaster* obtaining LC_50_s of 0.03 and 0.05 *μ*L/L, respectively [43]. Studies have shown that the *Eugenia uniflora* leaf (Pitanga) essential oil has toxicity against *D. melanogaster* at concentrations of 3 *μ*g/mL, 15 *μ*g/mL, and 30 *μ*g/mL, with mortality rates of 51, 79, and 78%, respectively [44].

Tests investigating the toxicity of the *Psidium guajava* (Goiaba) essential oil on *D. melanogaster* using the fumigation method found a significant increase in mortality, with this effect being associated with the time and concentration that the organism was exposed to, where the 23.5 and 30 *μ*g/mL concentrations presented the highest toxicity [45].

Toxicity assays evaluated through mortality and negative geotaxis are used as toxicity indicators of natural or synthetic chemicals, because they indicate through the mortality rate and damage to the locomotor apparatus physiological changes in the test organism, considering that the behavior is integrated to the subcellular and cellular processes of these organisms [46]. In addition, some studies in the literature perform biochemical assays to demonstrate physiological changes triggered by the substances in this alternative model, for example, we can cite oxidative stress as the main condition that is associated with the toxic profile of a substance, promoting an imbalance in the oxidant and antioxidant system of these organisms [47]. However, in this study, biochemical assays were not performed due to limitations in the technical facilities of the laboratory.

## 5. Conclusion

The present study demonstrated the reversal of resistance by efflux pump inhibition in *Staphylococcus aureus* carrying the TetK pump, which confers resistance to tetracyclines, by O-eugenol by ethidium bromide MIC reduction. Mortality and geotaxis assays with *Drosophila melanogaster* revealed the compound has moderate toxicity. This study is the first to analyze the antimicrobial activity of O-eugenol, as well as its toxicity. Investigating the mechanisms of action of natural compounds that present antibacterial effects by evaluating the gene expression profile is a fundamental requirement for drug discovery and development; however, due to technical limitations, these assays were not conducted in this study. Thus, future research should be encouraged to correlate gene expression in treated bacterial strains and possible molecular targets of the tested compounds.

## Figures and Tables

**Figure 1:** MIC of tetracycline in isolation and in combination with standard inhibitors and O-eugenol. CCCP: carbonyl cyanide m-chlorophenylhydrazone. ^∗^ represents statistical significance compared to the control.

**Figure 2:** MIC of ethidium bromide in isolation and in association with standard inhibitors and O-eugenol. CCCP: carbonyl cyanide m-chlorophenylhydrazone; ^∗^ represents statistical significance compared to the control.

**Figure 3:** *Drosophila melanogaster* mortality assays with the O-eugenol compound. ^∗^*p* < 0.05 compared to the control.

**Figure 4:** Negative geotaxis assays with the *Drosophila melanogaster* model.

**Table 1:** Minimum inhibitory concentrations of the associations between O-eugenol and standard inhibitors and ethidium bromide against the IS-58 *S. aureus* strain.

Substance	Control	Chlorpromazine	CCCP	O-eugenol
Tetracycline	128.0000	128.0000	25.39842	114.035
EtBr	32.0000	2.00000	16.0000	16.0000

EtBr: ethidium bromide; standard inhibitors: (CCCP) carbonyl cyanide m-chlorophenylhydrazone and chlorpromazine.

## Data Availability

The data will be available after request to the corresponding authors.
